The article "Clonal Analysis of Meningococci during a 26 Year Period Prior to the Introduction of Meningococcal Serogroup C Vaccines" was retracted in 2015. Reason: no approval from the institution.

# Clonal Analysis of Meningococci during a 26 Year Period Prior to the Introduction of Meningococcal Serogroup C Vaccines

**DOI:** 10.1371/journal.pone.0115741

**Published:** 2015-01-23

**Authors:** Christopher B. Sullivan, Mathew A. Diggle, Robert L. Davies, Stuart C. Clarke

**Affiliations:** 1 Scottish Haemophilus, Legionella, Meningococcus and Pneumococcus Reference Laboratory, Glasgow, United Kingdom; 2 Institute of Infection, Immunity and Inflammation, College of Medical, Veterinary and Life Sciences, University of Glasgow, Glasgow, United Kingdom; 3 Faculty of Medicine and Institute of Life Sciences, University of Southampton, Southampton, United Kingdom; 4 East Midlands Pathology, Clinical Microbiology Department, Queens Medical Centre, Nottingham University Hospitals NHS Trust, Nottingham, United Kingdom; University of Cambridge, United Kingdom

## Abstract

Meningococcal disease remains a public health burden in the UK and elsewhere. Invasive *Neisseria meningitidis*, isolated in Scotland between 1972 and 1998, were characterised retrospectively to examine the serogroup and clonal structure of the circulating population. 2607 isolates causing invasive disease were available for serogroup and MLST analysis whilst 2517 were available for multilocus sequence typing (MLST) analysis only. Serogroup distribution changed from year to year but serogroups B and C were dominant throughout. Serogroup B was dominant throughout the 1970s and early 1980s until serogroup C became dominant during the mid-1980s. The increase in serogroup C was not associated with one particular sequence type (ST) but was associated with a number of STs, including ST-8, ST-11, ST-206 and ST-334. This is in contrast to the increase in serogroup C disease seen in the 1990s that was due to expansion of the ST-11 clonal complex. While there was considerable diversity among the isolates (309 different STs among the 2607 isolates), a large proportion of isolates (59.9%) were associated with only 10 STs. These data highlight meningococcal diversity over time and the need for ongoing surveillance during the introduction of new meningococcal vaccines.

## Introduction

*Neisseria meningitidis* is an important cause of meningitis and bacteraemia worldwide. The UK has experienced a changing meningococcal epidemiology in recent decades, which may be due to the cyclical pattern seen in meningococcal serogroups as well as the implementation of meningococcal serogroup C (MenC) vaccines [1], [2]. A MenC immunisation programme was implemented in the UK in 1999. The vaccine was highly effective in reducing the incidence of serogroup C meningococcal disease and associated mortality, with no immediate adverse effects on other serogroups [3]–[5]. However, the natural history of meningococcal epidemiology is not well understood, particularly in relation to the long-term effect of MenC immunisation on the meningococcal population. It is therefore vital that the surveillance of meningococcal disease is continued. Long-term retrospective data is required as most contemporary information relates to immediately prior to or after the implementation of MenC vaccines. Although data is available on meningococcal serogroups dating back to the 1970s, and serogroup and serotype data is available from the 1990s, there is little molecular data available from the 1970s onwards. Using the collection held at the Scottish Haemophilus, Legionella, Meningococcus and Pneumococcus Reference Laboratory (SHLMPRL) from 1972 onwards, we describe the serogroup and clonal diversity of *N. meningitidis* in Scotland over several decades prior to the introduction of MenC vaccines.

The article "Clonal Analysis of Meningococci during a 26 Year Period Prior to the Introduction of Meningococcal Serogroup C Vaccines" was retracted in 2015. Reason: no approval from the institution.

## Materials and Methods

### Ethical approval

This work was carried out as part of routine public health investigations by the Scottish Haemophilus, Legionella, Meningococcus and Pneumococcus Reference Laboratory. The SHLMPRL is the national reference service for the detection and characterization of human Haemophilus, Legionella, Meningococcus and Pneumococcus infections and the identification and typing of associated environmental isolates. Patient consent was not required for this work. All data was anonymised and only bacterial isolates were used; no human tissue or clinical samples were used.

### Bacterial isolates

All isolates of *N. meningitidis* from blood, cerebrospinal fluid (CSF) and other normally sterile sites received by the SHLMPRL between 1972 and 1998 were included in the study. Isolates originated from patients with reported invasive meningococcal disease and were isolated at local diagnostic microbiology laboratories in all NHS regions across Scotland. Only one isolate was used per patient. Isolates were resuscitated from freeze-dried ampules in archive storage at the SHLMPRL by culturing on Columbia horse blood agar (Oxoid, Basingstoke, UK) and incubated overnight at 37°C in 5% CO_2_.

### DNA extraction

DNA was isolated as previously described [6] and used directly for PCR. For those freeze-dried meningococci that were not recoverable by culture, DNA was amplified directly from the freeze-dried vial.

### Isolate characterisation

Serogrouping was performed by latex agglutination when the meningococcal isolates were first submitted to the reference laboratory [7]. Those found to be non-groupable were characterised using *siaD* and *mynA* PCR as previously described [8]–[10]. Molecular characterisation was performed by multilocus sequence typing (MLST) based upon a semi-automated procedure [11]. The analysis of nucleotide sequence data and assignment of alleles and assignment of the allelic profile (otherwise known as the sequence type, ST) were performed as previously described [4], [12]. Clonal comparisons were made using eBURST2 [13].

The article "Clonal Analysis of Meningococci during a 26 Year Period Prior to the Introduction of Meningococcal Serogroup C Vaccines" was retracted in 2015. Reason: no approval from the institution.

## Results

### Serogroup characterisation

2607 isolates of *N. meningitidis* were available for analysis. 1434 were from CSF, 913 from blood and 260 from other sites (including skin scraping, joint aspirate, brain tissue, eye swab and rash fluid). There were 147 serogroup A isolates (5.6%), 1446 serogroup B isolates (55.5%), 812 serogroup C isolates (31.1%), 37 serogroup Y isolates (1.4%), 67 serogroup W isolates (2.6%), 10 serogroup X isolates (0.4%), five serogroup Z isolates (0.2%) and six serogroup E isolates (0.2%). Eighty-two isolates were initially non-groupable using latex agglutination but PCR reduced that number to 19 (0.7%). A further 58 isolates (2.2%) could not be characterised using either serogrouping or MLST by phenotypic or molecular methods. Serogroup distribution changed from year to year. Serogroup A meningococci were associated with 143 cases of invasive disease. The incidence of serogroup A was higher during the 1970s before declining substantially. 134 isolates (94%) occurred between 1973 and 1982, followed by three cases in 1986, two cases in 1987, one in 1989, one in 1992 and two in 1995. Serogroups B and C were the dominant serogroups during the 1980s and 1990s (Fig. 1). Serogroups Y, WI35, X, Z and E were also present in Scotland over this time period, representing only 4.8% of the total.

**Figure 1:** Distribution of invasive isolates associated with each serogroup, Scotland 1972-98.

### Clonal analysis by MLST

There were 309 different STs with ten accounting for 1562 isolates (59.9%). These were ST-11 (14.3%), ST-8 (14.2%), ST-41 (8.1%), ST-153 (5.4%), ST-1 (4.9%), ST-32 (3.9%), ST-33 (2.9%), ST-269 (2.5%), ST-334 (1.9%) and ST-60 (1.9%). The STs grouped into 31 distinct lineages, with 67 singleton types. There were 177 new STs which accounted for 253 (9.7%) isolates. The ST-8 complex was predominant, accounting for 567 isolates (21.7%) (Table 1). This was represented by 21 different STs, the predominant being ST-8 (369, 65.1%), ST-153 (a *gdh* locus variant of ST-8) (141, 24.9%), and ST-66 (a *fumC* locus variant of ST-8) (18, 3.2%).

**Table 1:** Association of STs with predominant clonal complexes from Scotland 1972–98.

Clonal complexes	Number of isolates	Number of different STs	STs present in double figures within clonal complex (%)				
ST-8	567	21	ST-8 (65.1%)	ST-153 (24.9%)	ST-66 (3.2%)		
ST-41/ST-44	422	51	ST-41 (49.7%)	ST-206 (12.1%)	ST-180 (6.4%)	ST-43 (5.2%)	ST-1362 (4.7%)
ST-11	393	12	ST-11 (95.1%)	-			
ST-32	239	21	ST-32 (42.7%)	ST-33 (31.4%)	ST-259 (8.0%)	ST-343 (6.3%)	
ST-1	133	5	ST-1 (96.2%)				
ST-269	132	26	ST-269 (48.5%)	ST-275 (24.2%)			
ST-334	107	23	ST-334 (49.5%)	ST-189 (14.0%)	ST-415 (12.1%)		

The article "Clonal Analysis of Meningococci during a 26 Year Period Prior to the Introduction of Meningococcal Serogroup C Vaccines" was retracted in 2015. Reason: no approval from the institution.

### MLST analysis by decade and serogroup

To determine the changes that might have occurred within the meningococcal population during the study period, analysis was performed by splitting the data into the time periods 1972–1979, 1980–1989 and 1990–1998, to fit with the suspected timing of the clonal expansion of MenC during the 1990s. Between 1972 and 1979 there were 616 isolates and these comprised 54 STs. There were 20 different clonal complexes and five singletons. Between 1980 and 1989 there were 845 isolates and these comprised 182 STs. There were 25 different clonal complexes and 39 singletons. Between 1990 and 1998 there were 1146 isolates comprising 160 STs. There were 27 different clonal complexes and 31 singletons.

The ST-8 complex was predominant during the 1980s and 1990s but declined from 1993 in line with an increase in ST11. The ST41/44 complex was the next most common during the 1980s and 1990s, two-thirds of which were serogroup B. he ST-11 complex became dominant during the 1990s which was associated with the specific emergence of serogroup C ST-11 meningococci and which coincided with a reduction in the ST-8 strains which had been predominant during the 1980s and early parts of the 1990s.

Serogroup B isolates could be differentiated into 218 different STs, comprising 20 distinct lineages with 54 singleton types. Three lineages accounted for 888 isolates. The ST-41/44 complex was predominant with 333 isolates (23.0%) and these were divided into 42 different STs.

Serogroup C isolates could be differentiated into 84 different STs, comprising 13 thirteen distinct lineages with 11 singleton types. Three lineages accounted for 664 isolates which represented 81.7% of all serogroup C isolates. The ST-11 complex accounted for the majority of isolates (328, 40.4%), these were divided into eight STs, 314 were ST-11 (95.7%), three were ST-2510, three were ST-4644, two were ST-3298 and ST-67, ST-2942, ST-3455 and ST-4677 were represented by a single isolate. The ST-8 complex accounted for 243 isolates (29.9%) and they were divided into nine different STs, 208 were ST-8 (85.6%), 15 were ST-66 (6.2%), and 13 were ST-153 (5.3%). Serogroup C was initially not associated with a particular clone but the major STs included ST-8, ST-11, ST-206 and ST-334.

Nine STs were associated with serogroup A meningococci (ST-1, ST-5, ST-60, ST-2002, ST-2174, ST-2152, ST-2517, ST-4570 and ST-4571). However, 88.7% of isolates were ST-1. Serogroup Y isolates could be differentiated into 10 different STs within three distinct lineages, with four singleton types. The ST-23 complex was predominant accounting for 19 (51.4%) isolates of which six were isolated in the 1970s, five in the 1980s and eight in the 1990s. Serogroup W isolates could be differentiated into 11 different STs within four distinct lineages, with two singleton types. The ST-11 complex was predominant with 42 isolates.

The article "Clonal Analysis of Meningococci during a 26 Year Period Prior to the Introduction of Meningococcal Serogroup C Vaccines" was retracted in 2015. Reason: no approval from the institution.

## Discussion

Our long-term, nationwide study has provided a unique insight into the molecular epidemiology of meningococci causing invasive disease within Scotland in the period 1972–1998. Using serogroup and MLST data we have described the clonal distribution of invasive meningococci prior to and during the emergence of MenC disease in the UK. Our data complements that described in other studies performed during the implementation of MenC vaccines [2], [4], [14], [15].

Serogroup distribution changed from year to year in Scotland during the time period 1972–1998, but serogroups B and C were dominant. Serogroup A was present within the 1970s and early 1980s but has not re-established itself as a major cause of meningococcal disease in the UK or elsewhere in Europe [16]. Serogroup B was the predominant serogroup throughout the 1970s and early 1980s until serogroup C became predominant during the mid-1980s. Although serogroup Y meningococcal disease was a rare cause of invasive disease in Scotland between 1972 and 1998 it is important that microbiologists are aware of its potential for increasing in incidence after the introduction of MenC vaccines [1].

Although there was diversity in the STs recovered between 1972 and 1998, ten of these STs accounted for more than half of the isolates from the study. There is extensive evidence for the persistence of particular genotypes among meningococcal disease isolates [17], [18] and similar observations have been made with other bacterial species [19]. In the present study, clonal complexes associated with seven lineages accounted for 1993 isolates (76.4%). Thus, although there were infections associated with novel STs, the majority of disease was associated with the same predominant disease-associated complexes that have been found worldwide and over a number of years [20], [21]. During the 1980s and 1990s, there was a noted diversity at the complex, ST and singleton levels but there was less diversity in the 1970s. However, these results should be treated with caution as there was a 27% increase in the number of isolates received at the reference laboratory between the 1970s and 1980s, and a similar increase between the 1980s and 1990s which may affect the reported meningococcal diversity.

The article "Clonal Analysis of Meningococci during a 26 Year Period Prior to the Introduction of Meningococcal Serogroup C Vaccines" was retracted in 2015. Reason: no approval from the institution.

A number of studies have been performed with collections of meningococci. For example, the EU-MenNet project analysed over 4000 European disease isolates from 18 countries for three years from 2000 to 2002 [21]–[23]. Although its findings were broadly similar to those of the present study, the isolates were from the time period around MenC vaccine implementation. With the increasingly widespread use of meningococcal polysaccharide and conjugate vaccines, one of the continuing epidemiological concerns is the effect of immunisation on serogroup replacement within the meningococcal population [24]. As the first meningococcal serogroup B vaccine has now been licensed in Europe and elsewhere [25], studies on meningococci from carriage and disease remain important in order to monitor circulating meningococcal serogroups.
